RETRACTED

# Synergistic Effect of Stereotactic Radiotherapy Combined with Karelizumab on Patients with Advanced NSCLC

**DOI:** 10.1155/2022/7875627

**Published:** 2022-03-08

**Authors:** Jiayou Guo, Jiayi Guo, Beibei Cheng, Xingbang Sun, Hongwei Zhang, Jianxin Ma

**Affiliations:** Department of Oncology, Lianyungang Oriental Hospital Affiliated to Xuzhou Medical University, Lianyun 222042, China

## Abstract

In this paper, synergistic effects of stereotactic radiotherapy (SRS) combined with karelizumab on the patients with advanced NSCLC have been analyzed through extensive experiments. For this purpose, 100 patients with advanced NSCLC in our hospital from December 2018 to December 2020 were selected and divided into control group and observation group. The control group was treated with SRS, while the observation group was treated with karelizumab at the same time. The data of age, gender, BMI, pathological type, and clinical stage were collected and recorded. After 3 months of treatment, the short-term efficacy of the two groups was evaluated according to RECIST solid tumor efficacy evaluation standard. Fasting venous blood of all patients before and 3 months after treatment was collected. The serum levels of matrix metalloproteinase-9 (MMP-9), cytokeratin 19 fragment (CY211), carcinoembryonic antigen (CEA), and vascular endothelial growth factor (VEGF) were detected by the enzyme-linked immunosorbent assay. The KPS score was used to evaluate the quality of life before and after treatment. The incidence of fatigue, diarrhea, and other adverse reactions were compared between the two groups. The patients were followed up for 3 years, and the survival of all patients was recorded. The total effective rate of the observation group was 50.00% (23/46), which was evidently higher than that (27.78% (15/54)) of the control group (*P* < 0.05). After treatment, the parameters of CY211, MMP-9, VEGF, and CEA in the two groups were evidently lower than those before treatment, and the parameters of CY211, MMP-9, VEGF, and CEA in the observation group were evidently lower than those in the control group after treatment (*P* < 0.05). After treatment, KPS parameters of the two groups were evidently higher than those before treatment, and KPS parameters of the observation group were evidently higher than those of the control group after treatment (*P* < 0.05). The 1-year, 2-year, and 3-year survival rates of the observation group were 95.64% (44/46), 89.13% (41/46), and 80.43% (37/46), respectively, and the 2-year and 3-year survival rates of the observation group were evidently higher than those of the control group (*P* < 0.05). SRS combined with karelizumab in the treatment of patients with advanced NSCLC has good curative effect, can evidently inhibit the angiogenesis and tumor growth and metastasis, can evidently improve the quality of life of patients, has a good synergistic effect, and can be widely used in clinic.

RETRACTED

## 1. Introduction

Lung cancer is a malignant lung tumor with a high incidence worldwide, with rapid disease progression, high mortality, and poor prognosis [1]. Non-small cell lung cancer (NSCLC) has the highest incidence, accounting for more than 80% of lung cancer [2]. Because the early course of lung cancer is hidden, most patients are already in the middle and late stages when they are diagnosed, and the effect of surgical treatment is poor [3]. Radiotherapy is one of the most important treatment methods for MSCLC. With the continuous development of radiological technology in recent years, stereotactic radiotherapy (SRS) has played an important role in the treatment of lung cancer [4]. Nguyen et al. [5] found that SRS had achieved good results in the treatment of stage I lung cancer and early multifocal primary lung cancer. However, the treatment effect of SRS for advanced NSCLC patients is poor, with a high incidence of adverse reactions and poor quality of life of patients. As an important immunosuppressive molecule, programmed cell death protein 1 (PD-1) can inhibit the autoimmune response by inhibiting the function of T lymphocyte and finally achieve the function of preventing the occurrence of autoimmune diseases [6]. Carrelizumab is an antibody to PD-1, which can block the PD-1 pathway and enhance the body's antitumor immunity. Marsh et al. [7] found that relizumab was effective in the treatment of solid cancers such as gastric cancer, nasopharyngeal cancer, and liver cancer. In this study, 100 patients with advanced NSCLC admitted to our hospital from December 2018 to December 2020 were taken as the observation objects, to analyze the synergistic effect of SRS combined with carrilizumab in patients with advanced NSCLC.

In this paper, synergistic effects of stereotactic radiotherapy (SRS) combined with karelizumab on patients with advanced NSCLC have been analyzed through extensive experiments. For this purpose, 100 patients with advanced NSCLC in our hospital from December 2018 to December 2020 were selected and divided into the control group and observation group. The control group was treated with SRS, while the observation group was treated with karelizumab at the same time. The data of age, gender, BMI, pathological type, and clinical stage were collected and recorded. After 3 months of treatment, the short-term efficacy of the two groups was evaluated according to RECIST solid tumor efficacy evaluation standard. Fasting venous blood of all patients before and 3 months after treatment was collected. The serum levels of matrix metalloproteinase-9 (MMP-9), cytokeratin 19 fragment (CY211), carcinoembryonic antigen (CEA), and vascular endothelial growth factor (VEGF) were detected by the enzyme-linked immunosorbent assay.

RETRACTED

The rest of this paper is arranged as given below.

In subsequent section, the proposed mechanism, i.e., synergistic effects of stereotactic radiotherapy (SRS) combined with karelizumab on the patients with advanced NSCLC, has been described in detail which is followed by extensive analysis of the experimental results and observations. Generalized discussion is provided in the second last section which is followed by an extensive summary of the proposed study.

## 2. Materials and Methods

### 2.1. Basic Materials

100 patients with advanced NSCLC admitted to our hospital from December 2018 to December 2020 were taken as the observation objects.

#### 2.1.1. Inclusion Criteria

1. All patients were diagnosed with NSCLC by pathological examination, confirmed by cytological and histological examination for three to four stages NSCLC
2. The serum indicators of the patient, such as white blood cells, neutrophils, and platelets were all in the normal range, and the expected survival time was ≥5 months
3. The patients and their family members were informed and signed the informed consent

#### 2.1.2. Exclusion Criteria

1. The patient was allergic to the experimental drug.
2. The patient's heart, liver, kidney, and other important organs had serious dysfunction.
3. The patient was mentally ill and could not cooperate with treatment.
4. The patient was complicated with other malignancies.
5. The clinical data of the patient was incomplete.
6. A history of chest radiotherapy, or pulmonary diseases such as atelectasis and pancreatic embolism pneumonia.
7. The patient refused the experiment or terminated the experiment for other reasons.

This experiment was approved by the hospital ethics committee.

### 2.2. Proposed Method

According to treatment methods, they were divided into the control group and observation group. Patients in the control group were treated with SRS, and patients in the observation group were treated with carrelizumab while receiving SRS.

Control group: the control group was asked to be in the supine position with arms crossed, and simulated positioning was carried out by CT with a layer thickness of 5 mm. Treatment range is as follows: the primary tumor and local metastases shown by CT, the displacement of respiratory movement in all directions as the gross tumor target (IGTV), and the planning target area (PTV). Radiological dose: IGTV was given 60 Gy/8F and 105 Gy bioavailable dose (BED), once a day, 5 times a week.

RETRACTED

Observation group: the SRS treatment was the same as the control group and received intravenous injection of carrelizumab, 200 mg/time, 28 days as a cycle, and treatment for 3 cycles.

### 2.3. Observation Index

Clinical information: the data of age, gender, BMI, pathological type, and clinical stage of the two groups were collected and recorded.

Short-term efficacy: CT examination was performed after 3 months of treatment, and the efficacy was evaluated using RECIST solid tumor efficacy evaluation criteria: disease progression (PD): the tumor size increased ≥25% or new lesions were found; no change (SD): the tumor size increased ≥25% or new lesions were found; partial remission (PR): the tumor size of lung cancer decreased ≥50%, duration ≥4 weeks; and complete remission (CR): the tumor tissue of lung cancer disappeared completely, and the duration was ≥4 weeks. Total efficacy = CR + PR.

Sera diagnosis: fasting venous blood from all cases before treatment and 3 months after treatment was collected and placed at room temperature for 20 min, centrifuged at 3000 r/min for 10 min, and put it in −70°C for refrigeration to avoid repeated freeze-thaw. Serum cytokeratin 19 fragment (CY211), vascular endothelial growth factor (VEGF), matrix metalloproteinase-9 (MMP-9), and carcinoembryonic antigen (CEA) were determined by the enzyme-linked immunosorbent assay.

Karnofsky performance scale (KPS) score was used to analyze the quality of life before and after treatment: KPS scores were obtained before treatment and 3 months after treatment, with a total score of 100. The higher the quality of life, the higher the KPS scores.

Adverse reactions: the incidence of adverse reactions, such as fatigue, diarrhea, pruritus, thrombocytopenia, and neutropenia were recorded and compared between the two groups.

Survival situation: the survival of all patients was recorded, and the follow-up period was 3 years.

### 2.4. Statistical Method

The data in this study were analyzed by the SPSS20.0 software package, enumeration data such as gender, pathological type, clinical stage, common efficiency of treatment, incidence of adverse reactions, and survival of each subject were expressed as percentage. *χ*^*2*^ was used for pairwise comparisons, serum CY211, MMP-9, VEGF, and CEA measurement data were expressed as (‾*x* ± *s*), pairwise comparisons were performed using the *t*-test. *P* < 0.05 was considered statistically significant.

## 3. Experimental Results and Observations

### 3.1. Comparison of Clinical Data between Two Groups

There was no significant difference in age, gender, pathological type, and clinical stage between two groups (*P* > 0.05). Comparison of clinical data between two groups is shown in Table 1:

RETRACTED

### 3.2. Comparison of Treatment Effect between Two Groups

The total effective rate of the observation group was 50.00% (23/46), which was evidently higher than 27.78% (15/54) of the control group (*P* < 0.05). Comparison of treatment effect between two groups is shown in Table 2:

### 3.3. Comparison of Serum Indexes between Two Groups

After treatment, the parameters of CY211, MMP-9, VEGF, and CEA in the two groups were evidently lower than those before treatment, and the parameters of CY211, MMP-9, VEGF, and CEA in the observation group were evidently lower than those in the control group after treatment (*P* < 0.05). Comparison of serum indexes between two groups is shown in Table 3:

### 3.4. Comparison of KPS Parameters of Two Groups

After treatment, KPS parameters of the two groups were evidently higher than those before treatment, and KPS parameters of the observation group were evidently higher than those of the control group after treatment (*P* < 0.05). Comparison of KPS parameters of two groups is shown in Table 4.

### 3.5. Comparison of Adverse Reactions between Two Groups

The incidence of adverse reactions in the observation group was 30.43% (14/46) and that in the control group was 22.22% (12/54), and there was no significant difference (*P* > 0.05). Comparison of adverse reactions between two groups is shown in Table 5:

### 3.6. Comparison of Survival between Two Groups

The 1-year, 2-year, and 3-year survival rates of the observation group were 95.64% (44/46), 89.13% (41/46), and 80.43% (37/46), respectively, and the 2-year and 3-year survival rates of the observation group were evidently higher than those of the control group (*P* < 0.05). Comparison of survival between two groups is shown in Table 6:

## 4. Discussion

The early stage of NSCLC is relatively secretive, unable to attract the attention of patients, and the course of the disease develops rapidly. It is often found in the middle and late stages. The treatment effect is not satisfactory and the patient's prognosis is poor [8]. SRS has been widely used in the treatment of advanced NSCLC patients with advanced age, poor lung function, and intolerance to surgery due to its advantages of noninvasive, short course of treatment, high target dose, and low peripheral normal tissue dose [9]. However, long-term SRS treatment can lead to different degrees of tolerance, increased incidence of adverse reactions, and poor quality of life in patients. PD-1 antibody has the advantages of long efficacy and few complications and is the focus of tumor immunotherapy related research in recent years. Shankar et al. [10] found that Carrelizumab treatment in advanced NSCLC patients could evidently improve the immune function of patients, which was of great significance in inhibiting the development of the disease. In this experiment, the total effective rate of recent treatment in the observation group was 50.00%, evidently higher than that in the control group (27.78%). The 1-year, 2-year, and 3-year survival rates of the observation group were 95.64%, 89.13%, and 80.43%, respectively. The 2-year and 3-year survival rates were evidently higher than those in the control group. SRS combined with carrilizumab in the treatment of advanced NSCLC patients had a good efficacy, had a good synergistic effect, and was of great significance for the effective treatment of patients.

RETRACTED

Cancer metastasis is the main cause of treatment failure in patients with advanced NSCL, and angiogenesis within the tumor plays an important role in cancer metastasis. CY211 is a marker produced during the apoptosis of alveolar epithelial cells. It is obviously highly expressed in lung cancer. The changes in its level reflect the changes in the condition of NSCLC [11]. CEA is evidently overexpressed in serum of patients with colon cancer, breast cancer, lung cancer, and other malignant tumors, and the decrease of its level can indicate the reduction of lung cancer tumor cells [12]. VEGF can induce the formation of new blood vessels of cancer cells and improve the infiltration ability of cancer cells by increasing vascular permeability. Xu et al. [13] found that the detection of VEGF had a certain value in predicting the metastasis of breast cancer cells. MMP-9 is a proteolytic enzyme that can degrade the vascular basement membrane and extracellular matrix components and participate in the metastasis of cancer cells. Liu et al. [14] found that MMP-9 could participate in the proliferation, metastasis, and invasion of gastric cancer cells by regulating the changes of VEGF indicators. In this study, after treatment, the levels of serum CY211, MMP-9, VEGF, and CEA in 2 groups were evidently decreased. The levels of serum CY211, MMP-9, VEGF, and CEA in the observation group were evidently lower than those in the control group. SRS combined with carrilizumab can evidently inhibit the formation of new blood vessels and the growth and metastasis of tumors, which was similar to the research results of Alidoosti et al. [15].

Extending the life cycle of patients and improving the quality of life of patients are the main clinical treatment principles for patients with advanced NSCLC [16]. KPS is a common score for evaluating the quality of life of patients, and it is widely used in clinical practice [17]. In this study, the KPS level of the observation group was significantly higher than that of the control group after treatment [18]. The adverse reactions of the two groups of patients were not statistically significant. SRS combined with carrelizumab in the treatment of advanced NSCLC was well tolerated and could effectively improve the quality of life of patients.

RETRACTED

## 5. Conclusion and Future Directions

In this paper, synergistic effects of stereotactic radiotherapy (SRS) combined with karelizumab on the patients with advanced NSCLC have been analyzed through extensive experiments. For this purpose, 100 patients with advanced NSCLC in our hospital from December 2018 to December 2020 were selected and divided into the control group and observation group. The control group was treated with SRS, while the observation group was treated with karelizumab at the same time. The data of age, gender, BMI, pathological type, and clinical stage were collected and recorded. After 3 months of treatment, the short-term efficacy of the two groups was evaluated according to RECIST solid tumor efficacy evaluation standard. Fasting venous blood of all patients before and 3 months after treatment was collected. The serum levels of matrix metalloproteinase-9 (MMP-9), cytokeratin 19 fragment (CY211), carcinoembryonic antigen (CEA) and vascular endothelial growth factor (VEGF) were detected by the enzyme-linked immunosorbent assay. In conclusion, SRS combined with karelizumab in the treatment of patients with advanced NSCLC has a good curative effect, can evidently inhibit the angiogenesis and tumor growth and metastasis, can evidently improve the quality of life of patients, has a good synergistic effect, and can be widely used in clinic.

## Figures and Tables

**Table 1:** Comparison of clinical data between two groups (‾*x* ± *s*).

Indicators		Control group (*n* = 54)	Observation group (*n* = 46)	*t/χ* ^*2*^	*P* value
Age		61.68 ± 5.46	62.74 ± 6.12	0.915	0.362
Gender	Male	32 (59.26%)	25 (54.35%)	0.245	0.621
	Female	22 (40.74%)	21 (45.65%)		
BMI		22.01 ± 1.08	21.74 ± 1.41	1.083	0.281

Pathological type	Adenocarcinoma	28 (51.85%)	22 (47.83%)	0.404	0.817
	Squamous carcinoma	21 (38.89%)	18 (39.13%)		
	Squamous adenocarcinoma	5 (9.26%)	6 (13.04%)		

Clinical stage	IIIa	6 (11.11%)	8 (17.40%)	0.881	0.643
	IIIb	29 (53.70%)	24 (52.17%)		
	IV	19 (35.19%)	14 (30.43%)		

**Table 2:** Comparison of treatment effect between two groups (n, %).

Groups	CR	PR	SD	PD	Total effective rate
Control group (*n* = 54)	0 (0.00%)	15 (27.78%)	20 (37.03%)	19 (35.19%)	15 (27.78%)
Observation group (*n* = 46)	0 (0.00%)	23 (50.00%)	15 (32.61%)	8 (17.39%)	23 (50.00%)
*χ* ^*2*^					5.206
*P* value					0.022

RETRACTED

**Table 3:** Comparison of serum indexes between two groups (‾*x* ± *s*).

Indicators		Control group (*n* = 54)	Observation group (*n* = 46)	*t*	*P* value
CY211	Before treatment	6.23 ± 2.06	6.38 ± 3.15	0.285	0.775
	After treatment	3.14 ± 1.85^a^	2.50 ± 0.85^a^	2.159	0.033

MMP-9	Before treatment	1856.39 ± 190.46	1874.23 ± 184.26	0.473	0.636
	After treatment	1524.39 ± 154.29^a^	1047.34 ± 80.16^a^	36.181	＜0.001

VEGF	Before treatment	749.68 ± 50.29	752.61 ± 54.69	0.278	0.780
	After treatment	469.38 ± 20.49^a^	265.49 ± 31.26^a^	39.090	＜0.001

CEA	Before treatment	21.95 ± 2.84	20.96 ± 3.15	1.652	0.101
	After treatment	15.24 ± 2.41^a^	9.46 ± 1.85^a^	13.270	＜0.001

^a^Compared with before treatment in the same group, *P* < 0.05.

**Table 4:** Comparison of KPS parameters of two groups ($\bar{x}$ ± *s*).

Groups	KFS		*t*	*P* value
	Before treatment	After treatment		
Control group (*n* = 54)	61.28 ± 9.41	71.46 ± 10.59	5.280	＜0.001
Observation group (*n* = 46)	60.29 ± 8.46	77.58 ± 10.46	8.716	＜0.001
*t*	0.549	2.896		
*P* value	0.548	0.005		

**Table 5:** Comparison of adverse reactions between two groups (*n*, %).

Groups	Fatigue	Diarrhea	Itchy skin	Thrombocytopenia	Neutropenia	Total incidence
Control group (*n* = 54)	7 (12.96%)	3 (5.56%)	1 (1.85%)	1 (1.85%)	0 (0.00%)	12 (22.22%)
Observation group (*n* = 46)	8 (17.39%)	2 (4.35%)	0 (0.00%)	3 (6.52%)	1 (2.17%)	14 (30.43%)
*χ* ^*2*^						0.870
*P* value						0.350

**Table 6:** Comparison of survival between two groups (n, %).

Groups	1-year survival rates	2-year survival rates	3-year survival rates
Control group (*n* = 54)	52 (96.30%)	39 (72.22%)	33 (61.11%)
Observation group (*n* = 46)	44 (95.65%)	41 (89.13%)	37 (80.43%)
*χ* ^*2*^	0.026	4.438	4.416
*P* value	0.869	0.035	0.036

## Data Availability

The data used to support the findings of this study are included within the article.
